# The complete mitochondrial genomes of two freshwater snails provide new protein-coding gene rearrangement models and phylogenetic implications

**DOI:** 10.1186/s13071-016-1956-9

**Published:** 2017-01-06

**Authors:** Xidong Mu, Yexin Yang, Yi Liu, Du Luo, Meng Xu, Hui Wei, Dangen Gu, Hongmei Song, Yinchang Hu

**Affiliations:** Key Laboratory of Tropical&Subtropical Fishery Resource Application & Cultivation, Ministry of Agriculture, Pearl River Fisheries Research Institute, Chinese Academy of Fishery Sciences, Xingyu Road1, Guangzhou, 510380 China

**Keywords:** Pulmonate, Mitochondrial genome, Gene order, Phylogeny

## Abstract

**Background:**

Mitochondrial (mt) genome sequences are widely used for species identification and to study the phylogenetic relationships among Gastropoda. However, to date, limited data are available as taxon sampling is narrow. In this study we sequenced the complete mt genomes of the freshwater gastropods *Radix swinhoei* (Lymnaeidae) and *Planorbarius corneus* (Planorbidae). Based on these sequences, we investigated the gene rearrangement in these two species and the relationships with respect to the ancestral gene order and assessed their phylogenetic relationships.

**Methods:**

The complete mt genomes of *R. swinhoei* and *P. corneus* were sequenced using Illumina-based paired-end sequencing and annotated by comparing the sequence information with that of related gastropod species. Putative models of mitochondrial gene rearrangements were predicted for both *R. swinhoei* and *P. corneus*, using *Reishia clavigera* mtDNA structure as the ancestral gene order. The phylogenetic relationships were inferred using thirteen protein sequences based on Maximum likelihood and Bayesian inference analyses.

**Results:**

The complete circular mt genome sequences of *R. swinhoei* and *P. corneus* were 14,241 bp and 13,687 bp in length, respectively. Comparison of the gene order demonstrated complex rearrangement events in Gastropoda, both for tRNA genes and protein-coding genes. The phylogenetic analyses showed that the family Lymnaeidae was more closely related to the family Planorbidae, consistent with previous classification. Nevertheless, due to the position recovered for *R. swinhoei*, the family Lymnaeidae was not monophyletic.

**Conclusion:**

This study provides the complete mt genomes of two freshwater snails, which will aid the development of useful molecular markers for epidemiological, ecological and phylogenetic studies. Additionally, the predicted models for mt gene rearrangement might provide novel insights into mt genome evolution in gastropods.

**Electronic supplementary material:**

The online version of this article (doi:10.1186/s13071-016-1956-9) contains supplementary material, which is available to authorized users.

## Background

The hyperdiverse pulmonate gastropods [1] contains the medically important clade Hygrophila, which comprises the freshwater families Acroloxidae, Chilinidae, Planorbidae, Lymnaeidae and Physidae [2]. Many of these freshwater snails are intermediate hosts for flatworm parasites and transmit infectious diseases of human and veterinary importance such as fascioliasis, cercarial dermatitis and schistosomiasis [3–5]. Accurate identification of species and analysis of genetic variation within populations is essential for studying molecular epidemiology and controlling parasite infection. However, previous studies suggest that pulmonate snails such as those of the genera *Radix* and *Planorbarius* exhibit a great diversity in shell morphology with extremely homogeneous anatomical traits [6]. Varying environmental factors seem to affect the morphological features resulting in variations and making it difficult to identify the species accurately on the basis of external features. Additionally, the evolutionary relationships among different molluscan classes and within some major clades are still unclear, due to the limited taxon sampling [7, 8].

Owing to the unique features such as maternal inheritance, lack of extensive recombination, a relatively high evolutionary rate and abundantly available marker types [6], mitochondrial (mt) genomes have been widely used for species identification, population genetics and evolutionary relationships studies in metazoans including pulmonates [4, 5, 8]. In general, the metazoan mt genome is a single circular DNA molecule of about 14–17 kb in size, typically containing 37 genes [9]: 13 protein-coding genes (PCGs) [cytochrome *c* oxidase subunits 1–3 (*cox*1-*cox*3), apocytochrome b (cyt*b*), ATPsynthase subunits 6 and 8 (*atp*6 and *atp*8), NADHdehydrogenase subunits 1–6 and 4 L (*nad*1-6 and *nad*4L)], two ribosomal RNAs [small and large subunit ribosomal RNA (rrn*S* and rrn*L*)] and 22 transfer RNA (tRNA). Typically, there are few non-coding regions containing repeat elements or pseudogenes, which are the usual source of size variations in metazoan mtDNA. With recent methodological advances, particularly the next generation sequencing technologies and the associated cost reduction in DNA sequencing [10], a growing number of complete mt genome sequences are available for mollusks in the GenBank database. Pulmonate snails like *R. swinhoei* and *P. corneus* are pathogen carriers and research into their basic biology has medical implications. *Radix swinhoei* serves as the major intermediate host of pathogens such as *Fasciola hepatica*, *Trichobilharzia paoi*, *T. physellae*, *T. ocellata*, *Echinostoma revolutum*, *E. hortense*, *Orientobilharzia turkestanicum*, *Angiostrongylus cantonensis*, *Cercaria ohiensis*, *Plagiorchis muris*, *Euparyphium ilocanum*, *Echinoparyphium recurvatum*, *Diplostomum niedashui* and *D. hupensis* in China, Japan, Thailand, India and Vietnam [3, 11]. *Planorbarius corneus* is the dominant intermediate host snail for the transmission of *Prosthogonimus ovatus*, *Apatemon gracilis, Hypoderaeum conoideum*, *Syngamus trachea* and *Typhlocoelum sisowi* worldwide [3, 12]. In this study, we used the Illumina-based paired-end sequencing [13] to report novel complete mt genomes of the freshwater snails *Radix swinhoei* and *Planorbarius corneus*, belonging to the families Lymnaeidae and Planorbidae, respectively. Mt gene rearrangement in pulmonate gastropods is of key interest to scientists from the perspective of understanding evolution and genome diversification. Further sequence analysis of the two snail species under investigation revealed novel gene rearrangements involving both protein-coding and tRNA genes. Together with other published complete mt genomes of heterobranchs gastropods, we reconstructed the phylogenetic relationship using the amino acid sequences of the 13 protein-coding genes with two different computational algorithms (maximum likelihood and Bayesian inference analysis). These data would provide valuable information not only for phylogenetic studies but also for the development of useful genetic markers for stock management and molecular epidemiological studies of parasites.

## Methods

### Specimen collection and DNA extraction

One adult individual of each *R. swinhoei* and *P. corneus* was collected from the Aquatic Invasive Risk Assessment Center, Pearl River Fisheries Research Institute Chinese Academy of Fishery Sciences (23°04′04.05″N, 113°13′06.97″E) in Guangzhou, Guangdong Province, China. The specimens were washed in physiological saline, identified morphologically according to existing descriptions of mollusc shape [3], fixed in 70% (v/v) ethanol and stored at -20 °C. Total genomic DNA was isolated from each species using approximately 30 mg of fresh foot tissue with OMEGA EZNA Mollusc DNA kit following the manufacturers’ instructions. Total DNA was eluted in sterile deionized water and was stored at -20 °C.

### Mitochondrial genomes sequencing, assembly and annotation

Paired-end libraries (500 bp) using TruSeq DNA Sample prep kit were prepared following the Illumina instructions. The size-selected, adapter-modified DNA fragments were PCR-amplified using PCR primers following the protocol: polymerase activation (98 °C for 2 min) followed by 10 cycles (denaturation at 98 °C for 30 s, annealing at 65 °C for 30 s, and extension at 72 °C for 60 s) with a final, 4 min extension at 72 °C. DNA libraries were purified by magnetic beads and quantified by real time quantitative PCR (RT-PCR).

Sequencing using Hiseq 2500 plate resulted in 1.23 Gb (*R. swinhoei*) and 1.44 Gb (*P. corneus*) high quality reads, containing 18,322 reads and 4514 reads of mitochondrion, respectively (Additional file 1: Table S1). Pair-End 100 bp read length of Illumina reads were analyzed. Reads that contained adapters were trimmed, and low quality reads which have more than 3 “N” base were removed. The first assembly using the chloroplast and mitochondrion assemble (CMA) V1.1.1 software (Guangzhou SCGene Co., Ltd) was based on overlap with the mt genomes of related species and paired-end relationships. The assembled complete mt genomes were tested for completeness and preciseness through paired-end read mapping back to the genome. For *P. corneus*, an uncertain region (nt 6275–6731) was amplified using the primers (F: 5′-ATG TGG GTT GTC AAT TAT CTG GT-3′; R: 5′-GCT ATA ACT AAG CTA TTG GGC TC-3′). The PCR reactions were prepared with a 40 μl total volume as follows: 20 μl 2× Taq master Mix (100 μmol/l) (GC gene), 2.0 μl of each primer (10 μmol/l), 15 μl ddH_2_O, and 1 μl DNA sample (0.2 ~ 0.5 μmol/l). The following PCR cycle was used for all fragment amplifications: an initial denaturation at 94 °C for 4 min; 35 cycles of 94 °C for 30 s (denaturation), 55 °C for 30 s (annealing), and 72 °C for 2 min (extension); followed by a final extension at 72 °C for 10 min. PCR products were examined using 1% agarose gel electrophoresis to validate the amplification efficiency and were sequenced using an ABI 377 (Applied Biosystems) automated DNA sequencer using the same primers (one primer at a time) as that for PCR. After *de novo* assembly and functional annotation, 13 protein-coding genes, rDNA genes, and tRNAs of mt genome were found, and compared with the two known complete mt genome of species of the family Lymnaeidae: *Galba pervia* (JN564796) [4] and *Radix balthica* (HQ330989) [14]. The related data were deposited in the National Center for Biotechnology Information (NCBI) Biosample databases with the accession numbers: SRS781941 (*R. swinhoei*) and SRS781939 (*P. corneus*). The two complete mt genomes were deposited in the GenBank database: KP279638 (*R. swinhoei*) and KP279639 (*P. corneus*).

### Sequence analysis

The complete mt genome sequence of *R. swinhoei* and *P. corneus* was aligned with other pulmonate complete mt sequences obtained from GenBank (Additional file 1: Table S2) by Clustal ×1.83 [15], using default parameters, and following the guidelines of the SeaView software [16]. Codon usage and nucleotide composition statistics were computed using Molecular Evolutionary Genetics Analysis (MEGA) 6 [17]. The protein-coding regions were identified by Basic Local Alignment Search Tool (BLAST; blastn, tblastx) from National Center for Biotechnology Information (NCBI) database and by using the MITOS WebServer BETA (http://bloodymary.bioinf.uni-leipzig.de/mitos/index.py) [18]. The transfer RNA genes were annotated using tRNA scan-SE v.1.21 (http://lowelab.ucsc.edu/tRNA scan -SE) with Search Mode = “Eufind tRNA- Cove”, Genetic Code = “Invertebrate Mito”, and Cove score cut-off = 0.1, and the software ARWEN (http://130.235.46.10/ARWEN/) [19]. The map of the species was visualized using the Genome Vx online tool (http://wolfe.ucd.ie/GenomeVx/) [20]. Repeat sequences were found using Spectral Repeat Finder v1.1 [21]. Strand asymmetry was calculated using the formulas: AT skew = (A-T)/(A + T) and GC skew = (G-C)/(G + C) [22]. Codon usage and building block distributions were determined gene-wise for all protein-coding genes, and merged using MEGA6.06 and statistical package R. Statistical analyses of distribution and codon usage heatmaps were generated using package R as well [23]. The stem-loop secondary structures of the non-coding regions were predicted using the default parameters under RNA folding option in the Mfold Server (http://www.bioinfo.rpi.edu/applications/mfold/) [24]. To conduct pair-wise comparison of the mt gene order of *R. swinhoei* and *P. corneus* with that of *Reishia clavigera* (name currently accepted for *Thais clavigera* [25]) as the standard gene pattern of molluscan mt genomes [26], we used CREx the program [27]. CREx is an efficient software suite which could analyze complex genome rearrangements scenarios in the gene order of a pair of taxa and determine the most parsimonious steps required for the rearrangement. In terms of rearrangement mechanism, the software can handle transpositions, reverse transpositions, reversals, and tandem duplication - random loss (TDRL) events among others. The analysis was performed by applying the common interval parameters for distance measurement and by using only protein-coding and ribosomal RNA genes. The more variable tRNAs were excluded from the analysis. Linear mt genome comparison of *R. swinhoei*, *P. corneus* and related species was performed using EasyFig2.1 (BLASTn, default setting) [28]. The graphical map was visualized with the CGView Comparison Tool (CCT) [29].

### Phylogenetic analyses

Phylogenetic analyses were performed using Bayesian inference (BI) and maximum likelihood (ML) methods. For the best-fit models of evolution for the amino acid sequence datasets (13 protein-coding genes) was selected ProtTest 2.4 [30]. BI was performed on combined database using MrBayes version 3.1.2 for 10,000,000 generations with a random starting tree. Four independent Markov chains were simultaneously run for ten million generations with a heating scheme (temp = 0.2) [31]. Trees were sampled every 100 generations (sample-freq = 100) with the first 25% of the generations were discarded as ‘burn-in’ and the remaining generations were used to compute the consensus tree. Stationarity was considered to be reached when the average standard deviation of split frequencies was below 0.01. ML analyses were conducted using PhyML 3.0 with 1000 bootstrapping based on the MtArt + I + G model [32]. The phylogenetic trees were drawn using the Evolview (http://www.evolgenius.info/evolview/#login) [33].

## Results and discussion

### Structural features of the mitocondrial genome

The complete mt genomes of *R. swinhoei* and *P. corneus* are 14,271 bp and 13,687 bp in length, respectively. The mt genome length of the two species of snail are comparable to that of other sequences of pulmonates (Additional file 1: Table S2). Mt genome of both *R. swinhoei* and *P. corneus* is a circular double-stranded DNA molecule, containing a total of 37 genes typically found in metazoans. These 37 genes belong to the following categories: 13 PCGs (*cox*1-3, *nad*1-6, *nad*4L, *atp*6, *atp* 8 and *cytb*), 1 *rrnS*, 1 *rrnL* and 22 tRNAs (Fig. 1). A high variation in nucleotide composition of pulmonate mt genomes has been reported [2, 4–6, 9, 14]. The variation of overall A + T content ranges from 54.76% (*Ovatella vulcani*) to 77.0% (*Succinea putris*), with an average value of 65.5% (Additional file 1: Table S2). The A + T content of *R. swinhoei* is 69.45% and of *P. corneus* is 72.66%, corresponding well with that of related species. The high A + T content is also reflected in the individual PCGs, with the values especially higher for *nad*6 gene (77.1%) for *R. swinhoei*, and *cox*2 gene (77.4%) for *P. corneus* (Adittional file 1: Table S3; Additional file 1: Table S4).

**Fig. 1:** Gene maps and organization of the complete mitochondrial genomes of *Radix swinhoei* (**a**) and *Planorbarius corneus* (**c**). The outer and the inner circles represent the positive (H-strand) and the negative (L-strand) strand, respectively. The tRNA genes are named using single-letter amino acid abbreviations as shown in the Tables (**b**, **d**). ^a^Indicates that the gene is encoded by H or L strand; ^b^ Intergenic nucleotides, indicates the number of nucleotides separating a gene from the one upstream of it; negative numbers indicate an overlap between the adjacent genes; ^c^Incomplete termination codon, which might probably be extended by post-transcriptional adenylation; ^d^Represent the presence of repeat masker

There are small variations in the AT- and GC-skews in pulmonate mt genomes. Due to the strand asymmetry (strand compositional bias) [34], the AT skews of the whole mt genome ranges from -0.210 (*Siphonaria gigas*) to -0.073 (*Albinaria caerulea*), while the GC skew values are between 0.047 (*P. corneus*) and 0.215 (*S. gigas*) (Additional file 1: Table S1). As with other pulmonate species, a similar AT and GC skews were detected in the mt genomes of both *R. swinhoei* and *P. corneus* (Additional file 1: Figure S1). Interestingly, the mt genome AT and GC skew values are similar between the two snails here studied. However, individual PCGs showed different and variable AT and GC skews in the *R. swinhoei* and *P. corneus* mt genomes (Additional file 1: Figure S2). AT skews were negative for most of the protein-coding genes except for *rrnS* (0.1) and *rrnL* (0.001) in *R. swinhoei*, and for *nad*2 (0.07) in *P. corneus*. On the other hand, GC- skews were positive generally, with negative values for *atp*6 gene (-0.1) in *R. swinhoei*, and for four genes, *atp*6 (-0.02), *cox*3 (-0.21), *rrnS* (-0.15); *rrnL* (-0.01) in *P. corneus* (Additional file 1: Table S3, Table S4, Figure S3). The nucleotide composition bias and skew may be caused by the selection-mutation-drift equilibrium of molecular evolution [35].

To better visualize the nucleotide identity in pulmonate mt genomes, we generated the graphical identity map using the CGView comparison tool (CCT). Taking gene order into account, an easy to track comparable graphic gene identity map was generated (Fig. 2). High conservation in the *cox* genes was observed with *cox*1 showing the highest similarity among several pulmonate species. On the other hand, *nad* genes were most variable with *nad*4L showing the maximal variation. Pairwise comparisons of the concatenated amino acid sequences revealed the overall mt genome similarity of 40.3–91.8% among pulmonate snails. This variation can be attributed to the rapid rate of mtDNA evolution.

**Fig. 2:** Graphical map showing nucleotide identity among the mitochondrial genes from *Radix swinhoei*, *Planorbarius corneus* and other pulmonate species. Gene specific identity was obtained by BLAST searches. The map is visualized by using the CGView comparison tool (CCT), which arranges BLAST result in an order where the sequence that is most similar to the reference (in this case *R. swinhoei*), is placed closer to the outer edge of the map

### Protein-coding genes (PCGs) and codon usage patterns

The full set of 13 PCGs, typically found in pulmonate species, were identified in the mt genome of *R. swinhoei* and *P. corneus*. Inferred initiation and termination codons from each protein-coding gene are shown in Fig. 1. Of the 13 PCGs, ten genes were found to initiate with the ATN codon, whereas three started with TTG in both *R. swinhoei* and *P. corneus.* These data are in accordance with previous findings from different gastropod clades [2, 4, 9, 14]. Most of PCGs were inferred to use TAA/TAG as stop codons except for T (*P. corneus*: *cox*1 and *cox*2), which frequently occurred in protein-coding genes of most gastropod mt genomes [5, 6, 8, 13]. The incomplete stop codon was thought to be complemented *via* post-transcription alpolyadenylation [36].

The various codon families and the Relative Synonymous Codon Usage (RSCU) for PCGs in *R. swinhoei* and *P. corneus* and their related species are summarized in Fig. 3. The total number of codons for all protein-coding genes in the mt genome of *R. swinhoei* and *P. corneus* were found to be 3443 and 3595, respectively (Additional file 1: Figure S4, Table S5, and Table S6). These numbers are distinctly small in comparison to that for *G. pervia* (3655) [4]. A bias towards T-rich codon was observed in the protein-coding genes, which may be attributed to the high percentage of Thymine in the mt genome of *R. swinhoei* and *P. corneus*. TTA coding for Leucine (Leu) was the most frequently used codon (203 times) in *R. swinhoei* (Additional file 1: Table S5) while TTT coding phenylalanine (336 times) was maximally represented in *P. corneus* (Additional file 1: Table S6). The codon families also exhibited a difference in their usage pattern among the two species, with Leu being the most frequent amino acid in *R. swinhoei* (16.94%) and Ser in *P. corneus* (11.10%) (Additional file 1: Figure S4). We also found a similarity in codon usage of *R. swinhoei* and *P. corneus* to that of the suborder Hygrophila. Although no major difference in codon usage was observed, the codons varied between different species and different genes. For example, a minor variation in the frequency of the codon TTA was observed among the investigated species.

**Fig. 3:** Codon usage distributions of all merged protein-coding genes among various pulmonate species. *Color key*: Color value around 1 (*green* region) implies that a codon was observed about 1 time in 60 codons indicating a uniform distribution. Higher (*red*) and lower (*blue*) values indicate deviations of uniform distribution (as factors). This map also helps us visualize the implicit variability in amino acid distribution. **a** Hierarchical clustering (average linkage method) of codon patterns (y-axis) approximately groups together the examined families. Closely related species (i.e., from the same tribe) generally have highly similar codon usage. Clustering of codon frequencies (x-axis) facilitates the visual identification of deviations. **b** The evaluation of relative synonymous codon usage

### Ribosomal and transfer RNA genes, and non-coding sequences

Similar to most of the other pulmonate mt genomes [4, 5], the location of *rrnL* is between tRNA-Val (V) and tRNA-Leu (L1), while that of *rrnS* is between tRNA-Glu (E) and tRNA-Met (M) in both *R. swinhoei* and *P. corneus* mt genomes (Fig. 1). The length of *rrnL* and *rrnS* in the *R. swinhoei* mt genome is 1370 bp and 827 bp and in *P. corneus* mt genome is 884 bp and 647 bp, respectively. The A + T contents of the rrn*L* and rrn*S* of both *R. swinhoei* (72.8 and 70.4%) and *P. corneus* (70.8 and 73.3%) were lower compared to that of *G. pervia* (*rrnL*: 74.93%; *rrnS*: 72.09%) [4]. Additionally, sequence alignment of *R. swinhoei* and *P. corneus* demonstrated sequence similarities for *rrnL* (67.6%) and *rrnS* (64.7%).

Both *R. swinhoei* and *P. corneus* contained 22 tRNA genes, ranging in size from 49 bp for both tRNA-Cys and tRNA-Glu (in *P. corneus*) to 75 bp for tRNA-Val (in *R. swinhoei*) with variations mainly arising from differences in stem and loop sizes of dihydrouridine (DHU) and TΨC. Most of the tRNA genes were predicted to have the typical cloverleaf secondary structure, except for tRNA-Gly (G), tRNA-Ser (S1) (AGN) and tRNA-Ser (S2) (UCN) in *R. swinhoei* (Fig. 4a), and tRNA-Cys (C), tRNA-Ser (S1) (AGN) and tRNA-Ser (S2) (UCN) in *P. corneus* (Fig. 4b). The tRNA-Gly (G) of *R. swinhoei* as well as tRNA-Cys (C) of *P. corneus* harbor a simple loop in the TΨC stem, while tRNA-Ser (S1) (AGN) and tRNA-Ser (S2) (UCN) of both *R. swinhoei* and *P. corneus* harbor a simple loop in the dihydrouridine (DHU) arm. Furthermore, tRNA rearrangements were predicted to occur in the *R. swinhoei* and *P. corneus* mt genomes. Such similar tRNA rearrangements have been reported in multiple divergent taxa, like *G. pervia* [4] and *R. balthica* [14].

**Fig. 4:** Analysis of possible secondary structure of mitochondrial tRNA genes and non-coding regions from *Radix swinhoei* and *Planorbarius corneus*. **a, b** Putative secondary structures of three representative tRNA genes identified in the mitochondrial genomes of *R. swinhoei* (**a**) and *P. corneus* (**b**); **c, d** Stem-loop secondary structures of two non-coding regions in the mt genomes of *R. swinhoei* (49 bp and 45 bp) (**c**) and *P. corneus* (112 bp and 71 bp) (**d**). Bars indicate Watson-Crick base pairings; dots indicate canonical base pairing between G and U nucleotides in RNA

As in most pulmonate snail species, both mt genomes contained a number of unassigned nucleotides, with the number ranging from 220 in *P. corneus* (1.6% of the genome) to 294 in *R. swinhoei* (2.1% of the genome). There are more than 30 non-coding regions throughout *R. swinhoei* (49, 45 and 36 bp in length) and *P. corneus* (112, 71 and 42 bp in length). The longest non-coding region (49 bp) in *R. swinhoei*, located between *cox*3 and tRNA-Ile gene, has a high A + T content (89.8%) and two stem-loop secondary structures (Fig. 4c), whereas the longest non-coding region in *P. corneus* (112 bp) lies between tRNA-Val and rrn*L* gene with a high A + T content (89.3%) and three stem-loop secondary structures (Fig. 4d). Although the functions of most of these non-coding regions remain unclear, the longest regions from both the species most likely are “putative control regions” owing to their sequence length and the presence of characteristic stem loop structure.

### Comparison of mitochondrial gene order

The gene order of the two mt genomes under investigation were compared to each other and to that of *R. clavigera* as a representative of the ancestral mollusc gene order within gastropods [26]. The gene order of the mt genomes of *R. swinhoei* and *P. corneus* is significantly different, with positional mismatches for both protein-coding and tRNA genes (Additional file 1: Figure S5). These findings are consistent with studies demonstrating high diversity in gene arrangements in pulmonate species, such as *G. pervia* [4] and *R. balthica* [14]. Some of the studies provide novel insights into the mechanism of mtDNA rearrangement in certain gastropod species [14, 37, 38]. Our results further support the view that tRNAs are involved in more frequent rearrangements than protein-coding genes and ribosomal DNA in metazoan mt genomes [38]. By comparing closely related species with different gene orders, the mt gene rearrangements could be usually explained by four possible models (the recombination model, tandem duplication and random loss (TDRL) model, tandem duplication and non-random loss (TDNL) model and tRNA miss-priming model) based on three mechanisms of gene arrangement (shuffling, translocation, and inversion) [39, 40]. However, for all rearrangement scenarios, tRNAs were not compared due to their higher variability in location.

We furthermore used the software CREx to reflect the genomic rearrangement history of *R. swinhoei* and *P. corneus*. The results effectively presumed that the gene rearrangement of *R. swinhoei* was postulated as follows. The first step was three times of continuous reversal: a reversal of 14 PCG genes except for *nad*5, a reversal of “*nad*4L-*nad*4” and a reversal of “*cox*2-*cox*1-*nad*1-*nad*2-*rrnL*” and “*Cytb*” (see three TDRL models in Fig. 5). Then, we performed the same analysis to presume the gene rearrangement form *R. clavigera* to *P. corneus*. The result showed that the first step was reverse transposition of *cox*2 gene. In the second of step, there were at least four putative reversals, including two reversals of 14 PCG genes except for *nad*5, a reversal of 13 PCG genes except for *nad*5 and *nad*6, a reversal of “*nad*3-*cox*3- *cox*2-*atp*6- *atp*8-*cox*1-*nad*2- *nad*1-*rrnL*-*rrnS*”. The third step included two TDRL. At last, there was a transposition of *rrnL* gene.

**Fig. 5:** Putative gene rearrangement events in gastropod mitochondrial genomes. *Reishia clavigera* was used as the standard ancestral gene pattern. Rearranged genes are indicated by different colors. Only the rearrangements for protein-coding and rRNA genes are taken into consideration. Four types of putative rearrangement events are possible in this context: reversal, reverse transposition, transposition and tandem duplication and random loss (TDRL). In the step-by-step scheme, the intermediate statuses are used to show different types of gene rearrangement events and the rearrangement process. **a** Putative gene rearrangement events from *R. clavigera* to *Radix swinhoei* mt genome. **b** Putative gene rearrangement events from *R. clavigera* to *Planorbarius corneus* mt genome

### Phylogenetic analyses

The phylogenetic relationships of pulmonate species based on concatenated amino acid sequence datasets using BI and ML analyses were reconstructed. The two 50% consensus trees had a similar topology with well-supported branches for major clades (Fig. 6). In the tree, all Panpulmonate species were clustered with high statistical support. Among the families represented by more than one species, the Helicidae, Planorbidae, Siphonariidae and Onchidiidae were recovered as monophyletic, while the Ellobiidae and Lymnaeidae were non-monophyletic due the recovered position of *Myosotella myosotis* and *R. swinhoei*, respectively. Some authors also recovered Ellobiidae as paraphylelic using the complete mt genomes [41–43] or partial genes [44], mainly due to the position of *Pedipes pedipes* or *M.myosotis*. Nevertheless, other phylogenies, such as those of Dayrat et al. [2] and Romero et al. [45] using nuclear and mt genes rendered Ellobiidae as monophyletic. Meanwhile, the taxonomic position of *R. swinhoei* should be revised. As pointed out by Lawton et al. [46] molecular identification was the only reliable method to identify *Radix* species and other Lymnaeidae since shell and other anatomical features are morphologically plastic and most species share morphological characters as a result of convergent adaptations to shared limnic environments.

**Fig. 6:** Phylogenomic analysis of concatenated proteins in mitochondrial genomes. The concatenated amino acid sequences of 13 protein-coding genes were analyzed utilizing Bayesian analysis (BI) and maximum likelihood (ML), using *Micromelo undata* and *Nautilus macromphalus* as the outgroup

The results also revealed that the families Lymnaeidae and Planorbidae are closely related with high statistical support, and the data obtained basically agreed with those of previous phylogenetic analyses based on complete mt genomes [4, 41–43, 47]. The taxa Sacoglossa (families Volvatellidae and Placobranchidae) and Siphonarioidea (family Siphonariidae) were recovered as sister clades, indicating closely relationships (already noted by Grande et al. [37]). Likewise, the Trimusculidae and Ellobiidae also showed sister-group relationships, previously pointed out by White et al. [47].

Additional complete mt genomes are needed for pulmonate snails (especially from missing lineages) in order to resolve the phylogenetic framework of this diverse group of gastropods to further understanding its evolution and obtain new information about the detailed processes and mechanisms of mt genome rearrangements.

## Conclusions

In this study, the characterization of the complete mt genomes of *R. swinhoei* and *P. corneus*, both encoding all the thirty-seven genes typical for pulmonates, revealed considerable interspecific differences in length and sequence composition. These genes were arranged in the same order as that of the proposed ancestral gastropod. However, the most remarkable feature was that, unlike in other pulmonate snails, a novel gene arrangement was observed. This study also provides an idea about novel mt genetic markers for species identification and population genetics of freshwater pulmonates and also has implications for the diagnosis, prevention and control of *Fasciola* spp. infection in hosts.

## Additional file

Additional file 1: Table S1. Summary of *Radix swinhoei* and *Planorbarius corneus* using Illumina sequencing. **Table S2.** General characteristics of the mitochondrial genomes of various members of pulmonate gastropods. **Table S3.** Nucleotide composition and AT- and GC-skews of the mitochondrial protein-coding and ribosomal RNA genes in the complete *Radix swinhoei* mt genome. **Table S4.** Nucleotide composition and AT- and GC-skews of the mitochondrial protein-coding and ribosomal RNA genes in the complete *Planorbarius corneus* mt genome. **Table S5.** Codon usage of *Radix swinhoei* mitochondrial protein-coding genes. **Table S6.** Codon usage of *Planorbarius corneus* mitochondrial protein-coding genes. **Figure S1.** Comparison of AT and GC skews among the 30 pulmonate species in Table S2. Circles and triangles separately represent AT and GC skews of the complete mitochondrial genomes. **Figure S2.** Gene specific strand composition of mitochondrial genome in *Radix swinhoei* and *Planorbarius corneus.* **Figure S3.** Graphical summary of nucleotide composition across complete mitochondrial genomes. **Figure S4.** Percentage of synonymous codon usage for each amino acid in *Radix swinhoei* and *Planorbarius corneus* mitochondrial protein-coding genes. **Figure S5.** Linear comparison of the gene distribution pattern of mitochondrial genomes between *Radix swinhoei* and *Planorbarius corneus*. (DOC 1430 kb)

## Abbreviations

ATP6 and ATP8: ATPase subunits 6 and 8
*cox*1-*cox*3: cytochrome *c* oxidase subunits1-3
*Cytb*: cytochrome *b*
ND1-ND6 and ND4L: NADH dehydrogenase subunits 1-6 and 4 L
NGS: Next-generation sequencing
PCG: Protein-coding gene
rRNA: ribosomal RNA
*rrnL*: Large rRNA subunit (gene)
*rrnS*: Small rRNA subunit (gene)
*trn*: Transfer RNA
